# Prediction of Hepatocellular Carcinoma Prognosis and Immune Cell Infiltration Using Gene Signature Associated with Inflammatory Response

**DOI:** 10.1155/2022/2415129

**Published:** 2022-01-07

**Authors:** Bin-Bin Da, Shuai Luo, Ming Huang, Fei Song, Rong Ding, Yao Xiao, Yang Fu, Yin-Shan Yang, Hai-Lei Wang

**Affiliations:** ^1^Department of Minimally Invasive Interventional Medicine Yunnan Cancer Hospital, Kunming 650118, China; ^2^CT Room, Kunming First People's Hospital, Kunming 650000, China; ^3^Hepatobiliary Pancreatic Vascular Surgery, Kunming First People's Hospital, Kunming 650031, China

## Abstract

It has been demonstrated that the inflammatory response influences cancer development and can be used as a prognostic biomarker in various tumors. However, the relevance of genes associated with inflammatory responses in hepatocellular carcinoma (HCC) remains unknown. The Cancer Genome Atlas (TCGA) database was analyzed using weighted gene coexpression network analysis (WGCNA) and differential analysis to discover essential inflammatory response-related genes (IFRGs). Cox regression studies, both univariate and multivariate, were employed to develop a prognostic IFRGs signature. Additionally, Gene Set Enrichment Analysis (GSEA) was used to deduce the biological function of the IFRGs signature. Finally, we estimated immune cell infiltration using a single sample GSEA (ssGSEA) and x-cell. Our results revealed that, among the major HCC IFRGs, two (DNASE1L3 and KLKB1) were employed to create a predictive IFRG signature. The IFRG signature could correctly predict overall survival (O.S) as per Kaplan-Meier time-dependent roc curves analysis. It was also linked to pathological tumor stage and T stage and might be used as a prognostic predictor in HCC. GSEA analysis concluded that the IFRG signature might influence the immune response in HCC. Immunological cell infiltration and immune checkpoint molecule expression differed in the high-risk and low-risk groups. As a result of our findings, DNASILE may play a role in the tumor microenvironment. However, more research is necessary to confirm the role of DNASE1L3 and KLKB1.

## 1. Introduction

Hepatocellular carcinoma (HCC) is the most frequent subtype of malignant hepatic cancer globally, accounting for 90% of all cases [1]. HCC is also the 5^th^ most frequent malignancy and the 3^rd^ most significant cause of cancer-related death worldwide [2, 3]. It has been suggested that hepatitis B and hepatitis C virus infection, alcohol abuse, and aflatoxin exposure are usually associated with HCC occurrence [4, 5]. Currently, despite tremendous advancements in HCC treatment options such as liver transplantation, chemotherapy, radiotherapy, and other potentially curative treatments, the long-term survival rate remains unsatisfactory due to the high likelihood of recurrence, with fewer than 20% of 5-year O.S rate [6, 7]. Luckily, the rapid development of gene sequencing technology offers some opportunities to unravel the molecular mechanisms of cancer [8, 9]. And ultimately resulting in that utilizing sequencing technology to screen the prognostic biomarkers and therapeutic targets of cancers has become prevalent. Nevertheless, the molecular mechanism of HCC occurrence and progression remains a challenge.

Increasing evidence has revealed that complex host inflammatory response is associated with the progression of cancers [10, 11]. Conversely, the inflammatory response may be a fundamental cause of nutrient and functional decline for patients with advanced cancer [12, 13]. On the other hand, the elevation of C-reactive protein levels introduced by inflammatory response was related to the compromised cell-mediated immunity, such as decreasing the number of lymphocytes, weakening T-lymphocytic response, and activating the innate immune system [14, 15]. More importantly, proinflammatory cytokines and growth factors involved in the inflammatory response may be related to tumor growth [10, 16]. Furthermore, there is evidence that the inflammatory response impacts the prognosis of certain tumors. C-reactive protein, for example, has been linked to the survival of non-small-cell lung cancer patients who have had resection [17, 18].

Meanwhile, C-reactive protein, albumin, and IL-6 are involved in non-small-cell lung cancer [19]. The upregulated C-reactive protein level in colorectal cancer can predict early recurrence and death [20, 21]. Besides, a recent study indicated that elevated C-reactive protein levels could predict the postoperative death of patients with liver metastases from colorectal cancer [22]. Furthermore, earlier research has linked C-reactive protein to the postoperative survival of HCC and perihilar cholangiocarcinoma patients [22, 23]. As a result, we hypothesized that inflammatory response-related genes (IFRGs) would be linked to HCC patients' overall survival.

Using data from The Cancer Genome Atlas (TCGA) database (https://tcga-data.nci.nih.gov/tcga/), we used weighted gene coexpression network analysis (WGCNA) and differential expression analysis to screen the important IFRGs in HCC patients in this study. Then, through the TCGA database and the GSE14520 dataset, a prognostic IFRG signature was created and verified. Finally, we looked into the relationships between the IFRG signature and the microenvironment of HCC.

## 2. Materials and Methods

### 2.1. Data Acquisition

The TCGA database was used to obtain the messenger RNA (mRNA) expression and clinical data of 50 normal and 374 primary HCC tissues (survival data was available for 374 HCC patients). Moreover, the GSE14520 dataset, containing 225 HCC patients (Survival information was available for 221 HCC patients) and 220 standard samples, which were sequenced by the GPL3921 platform, was obtained from the public Gene Expression Omnibus (GEO) database (https://www.ncbi.nlm.nih.gov/geo/) as a validation set. Furthermore, 773 IFRGs were obtained from the Molecular Signature Database v7.0”s “GOBP INFLAMMATORY RESPONSE” gene set (MSigDB, http://www.broad.mit.edu/gsea/msigdb/).

### 2.2. Construction of Weighted Gene Coexpression Networks

The *R* package “WGCNA” was used to perform weighted gene coexpression network analysis (WGCNA) [24]. Expression profile matrix of all genes (genes that are not expressed were removed) for 424 tissues in the TCGA database was used to perform WGCNA. Firstly, clustering of all samples was carried out to screen outliers. Then, using the results of Pearson correlation analysis between every two genes, the revised expression profile matrix of genes was converted into a similarity matrix, and the similarity matrix was changed into an adjacency matrix. Moreover, the scale-free topological algorithm selected the optimal soft threshold to ensure that the adjacency matrix met the scale-free topology criterion. Furthermore, the topological overlap matrix (TOM) and dissimilar TOM (dissTOM) were obtained based on the adjacency matrix's TOM similarity and dissimilarity. Finally, modules were screened using the Dynamic Tree Cut method by setting MEDissThres as 0.25 and minModuleSize as 50.

### 2.3. Identification of HCC-Related Module and Genes

Pearson correlation analysis was used to calculate the association between each module and samples' status to discover HCC-related modules and genes. A statistical correlation was defined as *P* < 0.05. Thus, the module with the highest positive or negative correlation with HCC was regarded as an HCC-related module, and genes in this module were preserved for further analysis.

### 2.4. Identification of Crucial IFRGs in HCC

To find key IFRGs in HCC, we used the *R* package “limma” to search the TCGA database for differentially expressed genes (DEGs) between HCC and normal samples [25]. The cut-off values were ∣log2 (fold change) | >1 and FDR < 0.05. Using the *R* packages “ggplot2” and “pheat map,” the volcano plot and heat map were created to display the expression levels of DEGs [26], respectively. In addition, overlapping genes among HCC-related genes, DEGs, and IFRGs were selected as key IFRGs by Venn diagram.

### 2.5. Correlations among Key IFRGs

Pearson correlation analysis was performed in the TCGA database to observe the correlations among key IFRGs based on their expression profile matrix. The *R* package “ggcorrplot” [27] was used to visualize the results of Pearson correlation analysis.

### 2.6. Construction and Validation of a Prognostic IFRG Signature

Using the “survival” package and the “step” function in *R*, univariate and multivariate Cox regression analyses were used to find prognostic IFRGs from the main IFRGs in the TCGA database to create a prognostic IFRG signature [28]. To illustrate the univariate and multivariate Cox regression analysis, the forestplots were drawn using the *R* package “forestplot.” The expression level and associated coefficient of prognostic IFRGs obtained from the multivariate Cox regression analysis created a prognostic IFRG signature. Each patient's risk value was computed as follows: (expression value of IFRG 1 coefficient of IFRG 1) + (expression value of IFRG 2 coefficient of IFRG 2) + ⋯ + (expression value of IFRG n coefficient of IFRG *n*) = risk value [29]. Thus, based on the median risk value, HCC patients in the TCGA database and the GSE14520 dataset were divided into high-risk and low-risk groups according to the risk value of each patient estimated using the formula mentioned above. Moreover, using the *R* package “survminer,” Kaplan-Meier (K-M) survival analyses and chi-square tests were used to assess overall survival (O.S.) between high-risk and low-risk groups. Furthermore, using the *R* package “survivalROC,” time-dependent receiver operating characteristic (ROC) curves were displayed to evaluate the IFRGs signature's prediction efficiency, and the area under the curve (AUC) for 1 year, 3 years, and 5 years O.S. was calculated [30].

### 2.7. Correlation between the IFRG Signature and Clinical Features

We used the Wilcoxon rank-sum test to evaluate the risk values in different clinicopathological characteristics (including age, gender, pathological tumor stage, pathological T stage, pathological N stage, pathological M stage, and child-pugh classification grade) in the TCGA database to see if there was a link between the IFRGs signature and clinical characteristics.

### 2.8. Independently Prognostic Analysis

To see if the IFRG signature and other clinical parameters could be employed as a stand-alone prognostic predictor, the independent predictive markers from the IFRGs signature (age, gender, pathological tumor stage, pathological T stage, pathological N stage, pathological M stage, and child-pugh classification grade) in the TCGA database were identified using univariate and multivariate Cox regression analysis. Furthermore, the results of univariate and multivariate Cox regression analyses were shown using the *R* package “forestplot,” with statistical significance defined as *P* < 0.05.

### 2.9. Gene Set Enrichment Analysis (GSEA)

GSEA was used to compare the biological functions of genes in high-risk and low-risk individuals. GSEA was performed using the expression matrix of genes between the high-risk and low-risk groups [31].

### 2.10. Assessment of the Immune Cell Infiltrating between the High-Risk and Low-Risk Groups

To determine if the IFRGs signature affects immune cell infiltration into the tumor microenvironment, we compared immune cell infiltration in the high- and low-risk groups in the TCGA database. First, we used a single-sample gene set enrichment analysis (ssGSEA) to assess the infiltration score of 16 immune cells and the activity of 13 immune-related pathways across high- and low-risk groups [32]. Furthermore, the infiltrating levels of anticancer immune cells and procancer immune cells were compared between the high-risk and low-risk groups using an *x*-cell algorithm [33]. In the tumor microenvironment, immune checkpoint molecules play a critical function. Thus, we also investigated several crucial immune checkpoint molecules (including BTLA, CD274, CTLA4, IDO1, IDO2, LAG3, PDCD1, and TIGIT) in the high-risk and low-risk groups.

### 2.11. Authentication of the IFRG Signature Genes' Expression Levels

Using the Wilcoxon rank-sum test, we first evaluated the mRNA expression levels of genes in the IFRGs signature between HCC and normal samples. Furthermore, the Human Protein Atlas (HPA, https://www.proteinatlas.org/) database was used to analyze the protein expression levels of genes in the IFRG signature.

### 2.12. Statistical Analysis

The *R* Studio was used for all of the statistical analyses in this study, and two groups were compared using the Wilcoxon test. The O.S. was compared between the high-risk and low-risk groups using a chi-square test. There was also a Wilcoxon rank-sum test run on HCC vs. standard samples to see any differences in gene expression in the IFRG signature between the two. When *P* was less than 0.05, the statistical analysis was significant even without specific instructions.

## 3. Results

### 3.1. Identification of HCC-Related Genes Based on WGCNA

Samples clustering identified 4 samples in the TCGA database as outliers (Figure 1(a)). As a result, a weighted gene coexpression network was built using the expression profile matrix of 420 samples from the TCGA database. By setting the ideal soft thresholds to 11 (scale-free *R*^2^ = 0.90, mean connectivity = 1), the scale-free topological algorithm revealed that the adjacency matrix met the scale-free topology criterion (Figure 1(b)). Moreover, 16 modules were screened by setting MEDissThres as 0.25 and minModuleSize as 50 (Figure 1(c)). Furthermore, correlation analysis of modules and samples status revealed that the MEmidnightblue module presents the highest correlation with HCC (*r* = 0.79, *P* = 1*e* − 92) (Figure 1(d)). Therefore, the MEmidnightblue module was defined as an HCC-related module, and 133 genes in the MEmidnightblue module were defined as HCC-related genes.

### 3.2. Identification of Crucial IFRGs in HCC

To identify key IFRGs in HCC, we firstly screened 4631 DEGs (including 4352 upregulated and 279 downregulated genes in HCC tissues compared to normal tissues) between HCC and normal tissues by setting the cut-off value as ∣log2 (fold change) | >1 and FDR < 0.05 (Figures 2(a) and 2(b)). In addition, a total of 12 overlapping genes (HAMP, TSLP, ESR1, KLKB1, FOS, ECM1, TBXA2R, CD5L, CCL14, DNASE1L3, CRHBP, and CCL23) among HCC-related genes, DEGs, and IFRGs were identified as crucial IFRGs in HCC (Figure 2(c), Table 1).

### 3.3. Correlations among Key IFRGs

We conducted the Pearson correlation analysis to observe the correlations among 12 key IFRGs further. As illustrated in Figure 3 and Table 2, all 12 key IFRGs showed a positive correlation. Moreover, DNASE1L3 displayed the highest positive correlation with CRHBP and CCL14 (Figure 3).

### 3.4. Construction and Validation of an IFRG Signature for Predicting the O.S. of HCC Patients

The TCGA database contained 374 HCC patients to create an IFRG signature based on 12 major IFRGs. As indicated in Table 3, a cut-off value of *P* < 0.1 was used to reserve DNASE1L3, KLKB1, CCL14, ESR1, CD5L, CRHBP, CCL23, and HAMP for multivariate Cox regression analysis based on the results of univariate Cox regression. Furthermore, an IFRG signature was created using the expression levels, and the associated coefficients of DNASE1L3 and KLKB1 were derived from the multivariate Cox regression analysis (*P* < 0.1, Table 4). Namely, risk value = (expression value of DNASE1L3 × (−0.0489)) + (expression value of KLKB1 × (−0.0065)). Therefore, each risk value of 374 HCC patients was calculated as the formula, and DNASE1L3 and KLKB1 acted as protective factors in HCC. We divided 374 HCC patients into the high-risk and low-risk groups according to the median risk value.

Furthermore, patients in the low-risk group lived longer than those in the high-risk group, according to K-M survival analysis (Figure 4(a)). According to ROC curves, AUC was 0.697 at 1 year, 0.67 at 3 years, and 0.63 at 5 years (Figure 4(c)). Furthermore, the patient survival status revealed that the high-risk group has more dead patients than the low-risk group (Figure 4(e)). Notably, with the increasing risk value, the expression levels of DNASE1L3 and KLKB1 decreased, which further indicated that both DNASE1L3 and KLKB1 acted as protective factors in HCC. Finally, we further validated the versatility and predictive efficiency of the prognostic IFRG signature in HCC samples in the GSE14520 dataset.

Similarly, the median risk values divided 221 HCC patients into high-risk and low-risk groups. We were surprised to see that the GSE14520 dataset matched the TCGA database's results (Figures 4(b), 4(d), and 4(f)). As a result, the IFRG signature based on DNASE1L3 and KLKB1 could accurately predict HCC patients' O.S.

### 3.5. Clinical Parameters and the IFRG Signature Correlations

There is a strong association between clinical features and the expression of the IFRGs signature in HCC. The IFRG signature was linked to the pathological tumor stage and T stage, as shown in Figure 5. HCC advancement may therefore be linked to the IFRG's signature.

### 3.6. In HCC, the Signature of the IFRG Was an Independent Prognostic Factor

We used the TCGA database to perform univariate and multivariate Cox regression analyses to uncover independent risk factors in HCC based on the FRG signature and clinical features. The univariate and multivariate Cox regression analysis results indicated that the IFRG signature was an independent risk factor for HCC patients, just as hypothesized (Figures 6(a) and 6(b)).

### 3.7. Identification of the IFRG Signature-Related Biological Function

The expression matrix of genes between the high-risk and low-risk groups in the TCGA database was utilized to perform GSEA to study the IFRG signature-related biological function. These genes were shown to be involved in metabolic pathways, PPAR signalling pathways, and immune-related biological processes, among other things (Figure 7). As a result, these findings suggested that the IFRG signature may play a critical role in HCC.

### 3.8. Correlations between the IFRG Signature and the Immune Cell Infiltrating in the Tumor Microenvironment

Based on the functional enrichment analysis results, we hypothesized that the IFRG signature would influence immune cell infiltration in the HCC microenvironment. As a result, we used the TCGA database to compare immune cell infiltration between high-risk and low-risk groups. ssGSEA suggested the enrichment scores of aDCs, APC co_ stimulation, check, consistent with our hypothesis. Cytolytic_activity, Mast_cells, macrophages, MHC_class_I, neutrophils, NK_cells, T_helper_cells, Treg, Type_I_IFN_Reponse, and Type_II_IFN_Reponse were significantly different between the high-risk and low-risk groups (Figure 8(a)). Significantly, the enrichment scores of macrophages, mast cells, NK cells, Type_I_IFN_Reponse, and Type_II_IFN_Reponse were the most statistically different between the high-risk low-risk group (Figure 8(a)).

Furthermore, the *x*-cell algorithm demonstrated that two anticancer immune cells (Th1 cells and CD4+ memory T-cells) and three procancer immune cells (Th2 cells, B-cells, and macrophages M2) distinguished the high-risk from the low-risk groups (Figures 8(b) and 8(c)). Furthermore, we investigated the relationships between the IFRG signature and immune checkpoint molecule expression levels. Most immune checkpoint molecules, including CTLA4, IDO2, LAG3, PDCD1, and TIGIT, were shown to be downregulated in the low-risk group compared to the high-risk group (Figure 8(d)). As a result, we hypothesized that the IFRG signature would influence HCC progression by controlling immune cell infiltration in the tumor microenvironment.

### 3.9. Validation of the Expression Levels of DNASE1L3 and KLKB1

To further confirm the potential roles of DNASE1L3 and KLKB1 in HCC, we further examined their expression levels in HCC patients. As expected, we found that both DNASE1L3 and KLKB1 are significantly downregulated in HCC tissues compared to normal tissues in the TCGA database and GSE14520 dataset (Figures 9(a) and 9(b)). Furthermore, immunohistochemical staining analysis using the HPA database revealed that the protein expression level of DNASE1L3 was downregulated in HCC tissues compared to normal tissues (Figures 9(c) and 9(d)). However, the HPA database did not identify any evidence of KLKB1 protein expression in HCC. Thus, DNASE1L3 and KLKB1 may play essential roles in HCC, but more research is needed to determine the roles of DNASE1L3 and KLKB1 in HCC.

## 4. Discussion

Each year, liver cancer is projected to cause over 600,000 deaths and 850,000 new cases worldwide [34, 35]. As the primary subtype of liver cancer, HCC has created a tremendous burden on society and has become an essential public health issue because of rapidly growing morbidity and mortality. Genetic and environmental factors affect the occurrence and development [36]. Several genes currently demonstrated an association with the tumorigenesis and progression of HCC, such as TP53 and CTNNB1, and can be used as the prognostic predictors of HCC [34]. Despite significant advances in treatment, the prognosis for HCC remains dismal due to the disease's significant heterogeneity [37, 38]. Thus, it is crucial to identify novel and more effective prognostic and therapeutic biomarkers in HCC. Currently, it has been established that the inflammatory response plays a crucial role in the carcinogenesis and development of HCC [39]. Hepatotropic viral infection, nonalcoholic steatohepatitis, and alcohol-induced fibrosis are all known to cause liver cancer through different processes [40, 41].

On the other hand, inflammation is a mechanism that all three of the disease as mentioned above processes share. Additionally, cytokines associated with the inflammatory response, such as IL2, IL5, and IL10, have been linked to the prognosis of HCC [42, 43]. However, due to the inflammatory response's complexity and multiplicity, the precise function of the inflammatory response in the progression of HCC remains unknown. This study created a predictive IFRG signature using two IFRGs (DNASE1L3 and KLKB1). Furthermore, we discovered that both DNASEILE3 and KLKB1 were downregulated in HCC tissues compared to normal tissues, with a higher expression indicating a better prognosis (Figures 4(e), 4(f), 9(a), and 9(b)). DNASE1L3, a member of the deoxyribonuclease 1 family, has been demonstrated to digest DNA in chromatin in both humans and mice and may be linked to autoimmune [44, 45]. Recent research has suggested that the overexpression of DNASE1L3 is involved in cancer cell death by degrading the tumor cell genome [46].

Moreover, the expression of DNASE1L3 can influence the progression of clear cell renal cell carcinoma [47]. DNASE1L3 has also been shown to alter the O.S in cancers of the colon, breast, kidney, liver, stomach, lung, sarcoma, and the prognosis of HCC patients after radical resection [48, 49]. Interestingly, DNASE1L3 is downregulated in HCC tissues relative to normal tissues. The higher expression of DNASE1L3 is associated with a better prognosis for patients with HCC [48, 50], which is consistent with our results. Our research has shown that DNASE1L3 can be used as a biomarker for HCC prognosis. Kinins and other vasoactive peptides are catalyzed by KLKB1 (also known as Fletcher factor), a glycoprotein encoded by KLKB1 [51]. Recent research has discovered that KLKB1 plays an essential role in forming bradykinin in several cancer types, including small cell lung cancer and prostate cancer, by participating in bradykinin formation [52, 53]. KLKB1 can be used as a diagnostic biomarker in chronic lymphocytic leukemia [54]. KLKB1 has not been explored as a predictive biomarker in tumors. As a result, our work is the first to discover that KLKB1 can be employed as a predictive biomarker for HCC.

It has been demonstrated that the inflammatory response is critical for immune function regulation. For instance, mounting evidence indicates that it is connected with weakened cell-mediated immunity [14, 55]. Nonetheless, the potential modification of the inflammatory and immunological responses remains a mystery. As a result, we investigated the relationship between IFRG signature and immune response. Surprisingly, the GSEA data indicated that immune-related biological processes were misaligned between the high-risk and low-risk groups (Figure 7). As a response, we examined differences in immune cell infiltration and immune checkpoint molecule expression between the high-risk and low-risk groups further.

Moreover, we found that most immune cell scores were markedly different between the high-risk and low-risk groups (Figure 8). Therefore, our study may contribute to understanding the correlation between inflammatory response and immune. Notably, the mutation of DNASEIL3 is involved in autoimmune diseases [56, 57]. More importantly, DNASILE3 can regulate immune response by activating neutrophils [15, 58] and multiple gene markers correlations of tumor-infiltrating immune cells, such as D.Cs, NK (natural killer) cells, neutrophils, and macrophages [50], which shows similarity to our results. Our study also found that neutrophils differed significantly between the high-risk and low-risk groups (Figure 8(a)). Therefore, our study further suggested that DNASILE may be necessary for the tumor microenvironment. In summary, we defined a novel prognostic IFRG signature to predict the O.S. of HCC based on 2 IFRGs (DNASE1L3 and KLKB1). In HCC, the IFRG signature can be used as an independent prognostic predictor. Additionally, the signature of IFRGs in HCC may impact the tumor microenvironment. Therefore, more research is needed to determine the role of DNASE1L3 and KLKB1.

## 5. Conclusion

Two of the main IFRGs in HCC (DNASE1L3 and KLKB1) were used to create a predictive IFRG signature. The IFRG signature can effectively and accurately predict overall survival (O.S.), as per Kaplan-Meier (K-M) time-dependent receiver operating characteristic (ROC) curves. Notably, the IFRG signature was associated with pathological tumor stage and pathological T stage, implying that it could be used as an independent prognostic predictor in HCC. Finally, GSEA analysis indicated that the IFRG signature would alter the immune response in HCC patients. Likewise, the quantity of invading immune cells and the expression of most immunological checkpoint markers differed significantly between the high-risk and low-risk groups. In this study, we created an IFRG signature to predict the prognosis of HCC. The IFRG signature was associated with invading immune cells, which could aid in HCC targeted therapy.

## Figures and Tables

**Figure 1:** The weighted gene coexpression network was constructed and screened HCC-related genes in the TCGA database. (a) Samples clustering to identify outliers. (b) Soft threshold selection analysis to select the optimal soft threshold. (c) A total of 16 modules were screened by setting MEDissThres as 0.25 and minModuleSize as 50. (d) MEmidnightblue module correlation with HCC.

**Figure 2:** Identification of crucial IFRGs in HCC from the TCGA database. (a) Volcano plot and (b) heat map presented the levels of expression of DEGs between normal tissues and HCC. (c) Venn diagram showing the overlapping genes among HCC-related genes, DEGs, and IFRGs.

**Figure 3:** The Pearson correlation analysis representations among 12 key IFRGs.

**Figure 4:** Construction and validation of the IFRG signature with two IFRGs in the TCGA database and the GSE14520 dataset. (a) Kaplan-Meier survival curves show the IFRG signature's prognostic value in the TCGA database and (b) GSE14520 dataset. (c) ROC curves depicting the prognostic, predictive efficiency for 1, 3, and 5 yr survival of HCC in the TCGA database and (d) GSE14520 dataset. (e) The expression profiles of DNASE1L3 and KLKB1, the risk score distribution, and patients' survival status in the TCGA database and (f) GSE14520 dataset.

**Figure 5:** Associations between the IFRG signature and TCGA database clinical features. (a)–(g) Distribution of the risk scores in different clinical characteristics: (a) age, (b) gender, (c) pathological tumor stage, (d) pathological T stage, (e) pathological N stage, (f) pathological M stage, and (g) child-pugh classification grade.

**Figure 6:** Illustrating the independent predictive analysis. (a) The results of univariate and multivariate analysis and (b) Cox regression analyses.

**Figure 7:** GSEA to investigate the IFRG signature-related biological function. (a)–(d) The result of KEGG pathway enrichment analysis. (a) propanoate metabolism, (b) pyruvate metabolism, (c) retinol metabolism, and (d) PPAR signaling pathway. (e, f) The immune-related biological process of G.O. enrichment analysis. (e) The somatic diversification of immunoglobulins and (f) somatic recombination of immunoglobulin gene segments.

**Figure 8:** Correlations between the IFRG signature and the immune cell infiltration in the tumor microenvironment. (a) ssGSEA algorithm compared the infiltrating score of 16 immune cells and the activity of 13 immune-related pathways between the high-risk and low-risk groups. (b, c) *x*-cell algorithm compared the infiltrating levels of anticancer immune cells (b) and procancer immune cells (c) between the high-risk and low-risk groups. (d) The expression levels of several important immune checkpoint molecules between the high-risk and low-risk groups.

**Figure 9:** Validation of the expression levels of DNASE1L3 and KLKB1. (a, b) DNASE1L3 and KLKB1 are significantly downregulated in HCC tissues compared to normal tissues in the TCGA database and (b) GSE14520 dataset. (c, d) The analysis of immunohistochemical staining from the HPA database.

**Table 1:** The expression levels of 12 key IFRGs in HCC.

Gene	conMean	treatMean	logFC	*p* value	FDR
HAMP	150.9095927	16.68886167	-3.176727057	3.10*E*-23	3.81*E*-22
TSLP	1.423747987	0.402100052	-1.824067374	1.55*E*-20	9.40*E*-20
ESR1	2.196110562	0.563842392	-1.961586832	6.25*E*-22	5.21*E*-21
KLKB1	58.47149021	27.55501713	-1.085418337	1.91*E*-17	7.17*E*-17
FOS	113.4523789	21.86418995	-2.375445056	2.38*E*-19	1.18*E*-18
ECM1	13.17346909	2.632176649	-2.323307095	1.38*E*-25	5.48*E*-24
TBXA2R	2.476759085	1.100354424	-1.170485253	5.80*E*-19	2.71*E*-18
CD5L	27.75172007	4.779279403	-2.537712176	3.56*E*-21	2.47*E*-20
CCL14	2.126415423	0.814094975	-1.385154455	6.80*E*-19	3.13*E*-18
DNASE1L3	26.29210932	4.823553659	-2.446461568	2.54*E*-24	4.84*E*-23
CRHBP	20.80654258	1.348160362	-3.947973234	8.68*E*-27	1.13*E*-24
CCL23	2.084707451	0.395844148	-2.396840513	2.37*E*-23	3.04*E*-22

**Table 2:** The correlations among 12 key IFRGs (*P* < 0.05).

	CCL14	CCL23	CD5L	CRHBP	DNASE1L3	ECM1	ESR1	FOS	HAMP	KLKB1	TBXA2R	TSLP
CCL14	1	0.5	0.4	0.5	0.8	0.4	0.4	0.3	0.4	0.3	0.5	0.4
CCL23	0.5	1	0.5	0.7	0.7	0.5	0.3	0.3	0.3	0.3	0.5	0.4
CD5L	0.4	0.5	1	0.6	0.6	0.4	0.3	0.3	0.4	0.2	0.4	0.3
CRHBP	0.5	0.7	0.6	1	0.8	0.7	0.5	0.5	0.5	0.4	0.6	0.5
DNASE1L3	0.8	0.7	0.6	0.8	1	0.7	0.5	0.4	0.5	0.4	0.6	0.5
ECM1	0.4	0.5	0.4	0.7	0.7	1	0.3	0.5	0.4	0.2	0.7	0.4
ESR1	0.4	0.3	0.3	0.5	0.5	0.3	1	0.3	0.2	0.5	0.2	0.4
FOS	0.3	0.3	0.3	0.5	0.4	0.5	0.3	1	0.2	0.3	0.4	0.4
HAMP	0.4	0.3	0.4	0.5	0.5	0.4	0.2	0.2	1	0.2	0.3	0.3
KLKB1	0.3	0.3	0.2	0.4	0.4	0.2	0.5	0.3	0.2	1	0.2	0.4
TBXA2R	0.5	0.5	0.4	0.6	0.6	0.7	0.2	0.4	0.3	0.2	1	0.3
TSLP	0.4	0.4	0.3	0.5	0.5	0.4	0.4	0.4	0.3	0.4	0.3	1

**Table 3:** Univariate Cox regression analysis identified the prognostic IFRGs.

Gene	HR	HR.95L	HR.95H
CCL14	0.58730961	0.395168728	0.872874175
CCL23	0.616922985	0.350249705	1.086636087
CD5L	0.860523195	0.756047244	0.979436371
CRHBP	0.77781906	0.621090565	0.974097054
DNASE1L3	0.714534334	0.611204635	0.835332858
ECM1	1.024482915	0.849411232	1.235638528
ESR1	0.614345839	0.423163278	0.891903504
FOS	1.015316807	0.910336986	1.132402873
HAMP	0.940656733	0.862436289	1.025971543
KLKB1	0.832497889	0.727817314	0.952234472
TBXA2R	0.858044327	0.607328164	1.212260704
TSLP	0.901955166	0.614808088	1.323214736

**Table 4:** Multivariate Cox regression analysis identified the optimal IFRGs to construct the IFRG signature.

Gene	HR	HR.95L	HR.95H
DNASE1L3	-0.04891162	0.952265287	0.916888259
KLKB1	-0.006514689	0.993506485	0.985980001

## Data Availability

The data used to support and substantiate the findings of this investigation are accessible upon request from the corresponding author.
